The article "Liability, risks, and recommendations for ultrasound use in the diagnosis of obstetrics diseases" was retracted in 2025. Reasons: unreliable results or conclusions; concerns about the citations.

# Liability, risks, and recommendations for ultrasound use in the diagnosis of obstetrics diseases

**DOI:** 10.1016/j.heliyon.2023.e21829

**Published:** 2023-11-04

**Authors:** Haiting Sun, An Wu, Minli Lu, Shan Cao

**Affiliations:** a Department of Ultrasound, The Affiliated Xiangshan Hospital of Wenzhou Medical University, Ningbo, 315700, Zhejiang Province, PR China; b Department of Obstetrics, The Affiliated Second People's Hospital of Yuhang District, Hangzhou City, Hangzhou, 311100, Zhejiang Province, PR China

**Keywords:** Misdiagnosis, Ultrasonography, Obstetrics, Pregnancy, Liability

## Abstract

This literature review will summarize the liability issues, risks, and ultrasound recommendations for diagnosing obstetrics diseases. One liability issue is related to misdiagnosis or failure to detect abnormalities during an ultrasound examination. Ultrasound images can be subjective interpretations, and errors may occur due to factors such as operator skill, equipment limitations, or fetal positioning. Another liability concern is related to the potential adverse effects of ultrasound exposure on both the mother and fetus. While extensive research has shown that diagnostic ultrasound is generally safe when used appropriately, there are still uncertainties regarding long-term effects. Some studies suggest a possible association between prolonged or excessive exposure to ultrasound waves and adverse outcomes such as low birth weight, developmental delays, or hearing impairment. Additionally, obtaining informed consent from patients is crucial in mitigating liability risks. Patients should be informed about the purpose of the ultrasound examination, its benefits, limitations, potential risks (even if minimal), and any alternative diagnostic options available. This ensures that patients know the procedure and can make informed decisions about their healthcare. Proper documentation helps establish a clear record of the care provided and can serve as evidence in any legal disputes.

## 1 Introduction

The use of ultrasound to diagnose and treat obstetric conditions has been vital for women's health. It provides essential diagnostic information quickly and at lower costs, and it is now standard equipment in almost all obstetric clinics globally. It is now the standard method for diagnosing pregnancy and other common obstetric problems [1]. However, there is considerable variation in the quality of available resources, including equipment, staff training, and even the interpreter's level of education and expertise. This may lead to incorrect diagnoses and interpretations. Inaccuracies in obstetric ultrasonography are a frequent cause of lawsuits, and this article discusses some ways litigation might be avoided. This literature review will summarize the liability issues, risks, and ultrasound recommendations for diagnosing obstetrics diseases. Conducting this review is crucial for ensuring patient safety, understanding legal implications, promoting evidence-based practice, driving quality improvement initiatives, and enhancing education and awareness among healthcare professionals.

The article "Liability, risks, and recommendations for ultrasound use in the diagnosis of obstetrics diseases" was retracted in 2025. Reasons: unreliable results or conclusions; concerns about the citations.

## 2 Methods

The design of the current investigation is a literature review that aims to discuss the liabilities and risks of using ultrasound in obstetric diseases. We conducted this study based on relevant published investigations and recommendations for review writing [2]. We performed a comprehensive search strategy to obtain as many relevant investigations and published protocols as possible. The searched databases include Web of Science, PubMed, Scopus, Google Scholar, and others. The following keywords were considered in the search strategy: (Liability OR Limitation OR risk OR misdiagnosis OR underdiagnosis OR thermal OR “Biological limitations” OR complications OR “adverse events” OR malpractice OR “informed consent” OR “image recording” OR “record-keeping” OR litigation OR “image acquisition” OR Errors OR mistakes OR interpretation OR perception OR communication OR education) AND (Ultrasound OR ultrasonography OR imaging) AND (obstetrics OR obstetric OR pregnant OR pregnancy). These terms were changeable and adapted based on each database's announced search guidelines.

### 2.1 Liability and risk of ultrasound in obstetrics

#### 2.1.1 Diagnostic errors

Overdiagnosis, underdiagnosis, and inaccurately reported test findings are all examples of diagnostic mistakes. A number of these incorrect diagnoses may be caused by artifacts introduced during the ultrasound examination's execution, namely in 2- and 3-dimensional ultrasonography during acquisition, processing, and presentation. Shadowing (which results in the “absence” of a structure) and reverberation (which results in the addition of a structure that is not there) are two of the most prevalent types of artifacts, although there are others that may occur when a reconstructed volume is manipulated, such as when a structure is deleted using an electronic scalpel [[3], [4], [5]]. A common kind of diagnostic error is the “invented” lesion, such as the appearance of a tumor when none exists or the lack of an organ or body part where the structure is otherwise healthy. These false-positive results might prompt unneeded diagnostic testing and even therapeutic interventions, such as abortion. An underdiagnosis occurs when an abnormality is only partly discovered, or not seen at all. For example, a false negative result could mean that a structural abnormality in the fetus was missed, a fetus was missed in a multifetal pregnancy, placental pathologies like placenta previa or accreta was missed, an ectopic pregnancy was missed because the pseudo sac was mistaken for the uterine cavity, or a mass was missed. Underdiagnosis may also include a diagnosis that is just partially correct.

The article "Liability, risks, and recommendations for ultrasound use in the diagnosis of obstetrics diseases" was retracted in 2025. Reasons: unreliable results or conclusions; concerns about the citations.

Misreporting includes but is not limited to, incorrect dating, incorrect estimated fetal weight, incorrect diagnosis (such as gender or presentation), failure to refer or perform a scan, miscommunication, lack of a formal report or error in report (“there was ventriculomegaly” when it should read “there was no ventriculomegaly”), and absence of documentation. Problems with underdiagnosis and reporting might aggravate conditions or result in the delivery of an abnormal fetus (which may be unwanted if the condition was known before birth) and subsequent legal action.

#### 2.1.2 Malpractice

The components of a malpractice claim are that 1) the provider owed the patient a duty of care, 2) the provider breached that duty (i.e., fell below the standard of care), 3) the patient suffered actual losses as a direct consequence of the breach, and 4) the provider's violation caused those actual damages to be compensable. In order to succeed in a liability case, all of the elements must be proven. Lawsuits involving health care are considered civil cases. Therefore, in a civil action, rather than having to show each element beyond a reasonable doubt, just a majority of the evidence (more than half) is needed. Inadequate image capture, mistakes in interpretation or reporting, and failure to get an imaging study are common points of emphasis in ultrasound-related litigation.

### 2.2 Informed consent

Informed consent requires both awareness and free will [6]. The reasonable person (patient) and reasonable physician criteria of consent are not uniform across the different guidelines and protocols. According to the reasonable patient standard, the information conveyed to a patient must be sufficient for the patient to be able to make an informed choice. According to the reasonable physician standard, a doctor in good standing would have given the patient the same information that was given to them. The permission form is only a memento of the patient and doctor's conversation and agreement that constitutes informed consent [6].

Ultrasound consent requires that the following topics be covered: 1) the diagnosis or nature of the problem, 2) the intended treatment, 3) choices of the procedure, including doing nothing, and 4) the significant hazards of the ultrasound or subsequent surgery. In addition, it is impossible to get fully informed permission without discussing the potential consequences of not doing an ultrasound [7,8]. The need for informed consent in writing for some types of ultrasonography tests varies by location and by institution. However, proper informed consent requires a discussion of the restrictions of any ultrasound investigation.

The article "Liability, risks, and recommendations for ultrasound use in the diagnosis of obstetrics diseases" was retracted in 2025. Reasons: unreliable results or conclusions; concerns about the citations.

For instance, obstetric ultrasonography presents a number of difficulties. There are three main obstacles to accurate fetal anatomy visualization: 1) the inability to see all deformities or anomalies, 2) the fact that certain anomalies change throughout the course of a pregnancy, and 3) the difficulties fetal position or mother body habitus imposes. Liability risks may be reduced by informing the patient of these restrictions and keeping a record of them. Moreover, including the patient's BMI in every ultrasound report is highly recommended. One of the most common problems with imaging is now solved in an objective way. It is also important to include in the written report whether there were any difficulties in seeing all the necessary anatomy to make a diagnosis. A consensus group on prenatal imaging has published recommendations for necessary follow-up in cases when fetal anatomy cannot be examined in its entirety [9,10]. If further appropriate visualization is not possible at the 2- to 4-week follow-up, a statement should be provided in the official report on these limits, and any subsequent tests should be guided by clinical indications. Limitations and lack of grounds for further ultrasound examinations should be communicated to patients.

Similarly, when a patient requests a gynecologic ultrasound, it is assumed that they provide their permission for the whole ultrasound to be performed. However, in cases of sonohysterography, sonosalpingography, or ultrasound-guided puncture, written verification of the patient's informed consent is required. Limiting legal risk requires talking about what can and can't be seen using vaginal and abdominal gynecologic ultrasonography. It is the main physician's responsibility to make any clinical-care choices based on the ultrasound results, thus the consulting sonologist should make that clear to the patient. That reasoning should presumably extend to transvaginal ultrasound as well. In most diagnostic units, however, it is not standard practice to have a chaperone present during sonographic exams performed by female sonographers and, on rare occasions, male sonographers. When men do transvaginal, vaginal, or rectal examinations, a chaperone is advised. All such examinations should provide patients with the option of a chaperone, and patients should provide verbal or written permission for the absence of a chaperone.

The article "Liability, risks, and recommendations for ultrasound use in the diagnosis of obstetrics diseases" was retracted in 2025. Reasons: unreliable results or conclusions; concerns about the citations.

### 2.3 The necessity of reporting and image recording

The American Institute of Ultrasound in Medicine (AIUM) has disseminated standards for reporting ultrasonography findings [11,12]. Best practices in ultrasound use are reflected in these recommendations, which specify what should be included in an ultrasound report and when. If major discoveries are not reported in a timely manner, an interpreting physician who deviates from the recommendations may be put in jeopardy. Each inspection should be documented formally with suitable picture documentation. A written report is preferable to a simple notation in the patient's file because it lends more authority to the laboratory or institution that performed the test and provides more detail to the referring doctor. Images must be kept for the length of time required by the statute of limitations in each state or jurisdiction in which they were created. Images are better preserved in a picture archiving and communication system (PACS) or digital format rather than thermal printouts.

### 2.4 Poor maintenance of equipment

Ultrasound technology has advanced at an exponential rate. Nowadays, most hospitals and clinics can afford high-quality medical equipment. Therefore, patients should anticipate that the facility would employ up-to-date, well-maintained equipment. When a medical facility continues to use outdated equipment that the manufacturer no longer maintains, it raises questions about the quality of treatment being offered. Poor image quality can increase the liability risk for doctors and their practices if preventative maintenance is neglected.

### 2.5 Supervision requirements

General, direct, and personal supervision are the three tiers of imaging study supervision. The doctor's physical presence is optional as long as the procedure is carried out under general supervision. However, the physician is responsible for educating the non-medical staff who does the diagnostic process and maintains the equipment. If the procedure is to be performed under the doctor's supervision, they must be present in the same office and readily available to offer aid and guidance at all times. However, the doctor's physical presence in the room where imaging is conducted is optional. When a procedure calls for the doctor's personal supervision, they must be present in the room at all times. Percutaneous umbilical blood collection, chorionic villus sampling, amniocentesis, and sonohysterography/sonosalpingography are the only obstetric/gynecological ultrasound procedures that require direct supervision [13,14]. Increased liability concerns and allegations of fraudulent billing may be brought against doctors when monitoring is inadequate.

The article "Liability, risks, and recommendations for ultrasound use in the diagnosis of obstetrics diseases" was retracted in 2025. Reasons: unreliable results or conclusions; concerns about the citations.

### 2.6 Incomplete or inadequate studies

Adequate images for diagnosis should be included in ultrasound investigations. Liability rises, in particular for missed diagnoses, when surveys are inadequate. When conducting an obstetric survey, researchers should follow the standards set by the AIUM and the American College of Obstetricians and Gynecologists (ACOG) [15,16]. This includes obtaining the necessary images for the study, using appropriate measurement criteria, and documenting the results correctly. Ultrasound studies benefit more from and are less risky when conducted in accordance with such standards. For instance, the cardiac outflow pathways are evaluated as part of the usual obstetric ultrasound assessment. A dating ultrasound, for example, does not provide the same information as a full obstetric ultrasound. A full anatomic survey, which is part of the routine obstetric ultrasonography, should be conducted as soon as possible in such cases. Patient referral for “targeted” or “detailed” ultrasound is warranted if more assessment is required after antepartum screening or ultrasound [16,17]. Inadequate surveying raises the likelihood that serious prenatal abnormalities may be missed, as well as the likelihood that serious legal consequences will result.

### 2.7 Exceptions for specific or targeted assessments

In 2009, the AIUM and the American Society for Reproductive Medicine (ASRM) published a consensus statement stating that nurses with ultrasound training and appropriate physician supervision can perform ultrasounds for follicular monitoring [18,19]. The group agreed that a thorough ultrasound scan within the previous 4–6 months was necessary to rule out serious gynecologic abnormalities.

### 2.8 Improper acquisition of images

Obtaining acceptable photographs is a crucial component of litigation in this field. This includes but is not limited to, the following issues: 1) inadequate training of the sonographer performing the ultrasound investigation, 2) an insufficient or incomplete study, with images of insufficient quality to make an appropriate diagnosis, 3) insufficient supervision of the sonographer, and 4) inadequate maintenance of the imaging equipment. Quality ultrasonic studies can be conducted according to the recognized standards. Accreditation can only be granted to practice if those requirements are completed. Accreditation of this sort demonstrates an organization's adherence to industry “best practices” and may strengthen its legal position should a lawsuit ever be filed [20].

### 2.9 Sonographer training

To ensure that sonographers are competent in study performance and image capture, they are subjected to rigorous training, testing, and certification. Sonographers working in hospitals must hold certification from an agency recognized by the American National Standards Institute-International Organization for Standardization or the National Commission of Certifying Agencies in order to be employed, per regulations set forth by the Joint Commission. The American Registry for Diagnostic Medical Sonography and the American Registry for Radiologic Technologists are both credible authorities that have earned accreditation. In the past, it was usual for ultrasound technicians to learn on the job without any sort of certification, but now, this is almost unheard of because of the increased importance put on formal education [21].

The article "Liability, risks, and recommendations for ultrasound use in the diagnosis of obstetrics diseases" was retracted in 2025. Reasons: unreliable results or conclusions; concerns about the citations.

### 2.10 Litigation-inducing errors

Liability cases against doctors typically involve one or more of the following categories of mistakes: incorrect perception, incorrect interpretation, failure to recommend the next best course of action, and failure to relay important results to the referring doctor [[22], [23], [24]].

### 2.11 Errors of communication

When performing or interpreting ultrasounds on referral, sonologists have a responsibility to share any important results with the referring physician. While a written report detailing the findings of an imaging investigation or operation is generally seen as the gold standard, there are times when verbal or in-person communication is required [25]. If a serious fetal abnormality is found, for instance, the referring doctor should be informed immediately and the conversation should be recorded in the final report. If the interpreting doctor does not rely on the results of the tests in a timely way that makes clinical sense, they might be held liable for wrongful birth [24]. Another case in point is when it is necessary to adjust a due date owing to pregnancy. When a patient has an elective delivery (such as a repeat cesarean), and the suggestion to move the due date up or down is not made explicit in the final report or conveyed to the referring physician, culpability may be claimed. The same holds true if a patient is diagnosed with an ectopic pregnancy but the news is not immediately relayed to the referring doctor. Subsequently, the patient may need emergency surgery, lose a fallopian tube, or perhaps die.

### 2.12 Errors of interpretation

When an anomaly is noticed but the description is wrong, an interpretation mistake usually occurs. A malignant tumor termed benign and a normal variation labeled abnormal are two examples. The former might include, for instance, a mucinous adenocarcinoma of the ovary that has been misdiagnosed as a dermoid. For instance, a bleeding corpus luteum might be misdiagnosed as a malignant tumor, leading to unneeded and invasive surgery. The best line of defense is a thorough differential diagnosis that includes the actual diagnosis, along with sensible suggestions for further testing (such as an endometrial biopsy or the acquisition of tumor markers). These situations are substantially more defendable when such advice is provided, with over 75 % correct interpretations when approached [19,26]. Litigation is on the rise when a misdiagnosed intrauterine pregnancy is treated with methotrexate as though it were an ectopic pregnancy [[27], [28], [29], [30], [31]]. The chance of miscarriage increases after using methotrexate, and the risk of fetal abnormalities increases if the pregnancy continues [32].

The article "Liability, risks, and recommendations for ultrasound use in the diagnosis of obstetrics diseases" was retracted in 2025. Reasons: unreliable results or conclusions; concerns about the citations.

Pregnancy of Unknown Location (PUL) should be the diagnosis when an ectopic pregnancy or an intrauterine pregnancy cannot be confirmed by the first ultrasound [33,34]. Ultrasound and serial hCG levels are recommended for monitoring. An ectopic pregnancy may be considered when hCG levels are excessively high but cannot be confirmed in isolation [[35], [36], [37], [38]]. Due to the presence of discriminating levels, extreme caution is warranted when ruling out an intrauterine pregnancy with rising hCG. According to the available research, the lack of an intrauterine gestational sac cannot be confirmed until the hCG level is over 2500–3500 mIU/mL [[39], [40], [41]]. When expecting more than one child, further caution is needed since even with high hCG levels, it is not always possible to identify an intrauterine gestational sac. Important precedents have been set in such situations.

### 2.13 Errors of perception

A perception error happens when a study's anomaly is later discovered. For instance, the interpreting doctor could have missed a fetal abnormality that was visible on the scans. When a patient claims to have an abortion if being aware of the anomalies before giving birth, this is an example of a wrongful birth claim [[42], [43], [44]]. Experts determine if the doctor's failure to notice the anomaly falls below the accepted level of care [45,46]. Such mistakes are hard to defend, and approximately eighty percent of cases that reach a jury verdict are lost [[45], [46], [47]]. Because of the potential for extremely large judgments at trial, lawsuits involving missed diagnoses are sometimes resolved out of court. A cancerous tumor that was first undetected by ultrasonography is another example. Patients' life expectancies are said to be shortened because of the increased severity of their condition at the time of diagnosis, decreased likelihood of recovery, and worsened prognosis as a result of the delay.

The article "Liability, risks, and recommendations for ultrasound use in the diagnosis of obstetrics diseases" was retracted in 2025. Reasons: unreliable results or conclusions; concerns about the citations.

### 2.14 Failure to recommend the next relevant procedure

An observant sonologist will provide recommendations for follow-up studies or procedures depending on the patient's current condition. For instance, if there is a large size disparity between the expected and actual due dates, it is advised that the due date be moved forward and confirmed by subsequent ultrasound exams. Interpreting sonologists will typically suggest repeated hCG readings, with a repeat ultrasound if clinically necessary, when an ectopic pregnancy might be present but the diagnostic findings are inconclusive. Similarly, if an endometrial thickness >4 mm is seen during ultrasound screening for postmenopausal bleeding, additional investigation, such as sonohysterography, hysteroscopy, or endometrial biopsy, should be recommended.

### 2.15 Neglecting an ultrasound

There are circumstances in which a Current Procedural Terminology (CPT) code 76811 is warranted in the field of obstetrics [48,49]. If a potentially diagnosable disease or abnormality may have been recognized, the practitioner runs a higher risk of responsibility if they fail to recognize these signals and do not send the patient for more advanced testing. Therefore, in order to mitigate potential legal consequences, it is essential for a provider to recognize individual risk factors and refer a patient without delay. If the physician fails to order the right tests while a patient is showing symptoms, they might face further legal trouble. Ovarian cancer symptoms include but are not limited to, recurrent complaints of stomach bloating and early satiety in a menopausal patient for >13 months or >1 year [50,51]. A diagnostic ultrasound, or referral to a specialist who can perform one, is essential in such situations.

The liability risk associated with delaying an ultrasound or imaging scan is high if the patient is later diagnosed with ovarian cancer. It is critical to patient treatment to determine whether or not an adnexal lump is cancerous and requires referral to a gynecologic oncologist. Recent recommendations from an international consensus panel state, “It is appropriate to consider referral to an expert gynecologic sonologist when faced with a challenging or indeterminate adnexal mass.” [52,53] A doctor's liability would rise if he or she failed to recommend a patient for such tests.

### 2.16 Biological risks

Since ultrasound is a sound wave—a kind of energy with alternating positive and negative pressure—the impacts on living organisms must be taken into account whenever the topic is explored. As a result, it has the potential to cause a wide range of changes (or “bioeffects”) in the tissues it passes through. Potentially harmful effects on tissues may be broken down into two categories: thermal and non-thermal (or mechanical) [[54], [55], [56], [57], [58], [59]]. The conversion of acoustic energy into heat is an indirect cause of thermal effects caused by the propagation of a waveform. This is the primary risk to developing embryos and babies [[60], [61], [62], [63]]. Animal research using both non-ultrasound and ultrasound technologies has shown that maternal heat exposure is hazardous to the developing embryo/fetus [60,[64], [65], [66], [67], [68], [69], [70]]. It seems to be the case if the temperature increases by more than 1.5 °C over the physiological threshold. Damage potential rises with both exposure time and concentration, and the developing embryo/fetus is especially vulnerable to external insult in the first 10–12 weeks of pregnancy. However, organ development continues well into the second trimester, and subtle changes in behavior, if they exist at all, are difficult to detect.

The article "Liability, risks, and recommendations for ultrasound use in the diagnosis of obstetrics diseases" was retracted in 2025. Reasons: unreliable results or conclusions; concerns about the citations.

Moreover, direct effects of the alternating pressure include non-thermal mechanisms such as acoustic cavitation (inertial and non-inertial), acoustic radiation torque (causing rotation or spinning in the insonated tissue), acoustic radiation force (time-averaged force exerted by the ultrasound beam), and acoustic streaming (circulatory flow). It seems that non-thermal processes are not a significant cause for worry when using ultrasonography for obstetrics [[71], [72], [73]]. Since cavitation requires the existence of cavitational foci (bubbles), which are not present in the fetal lungs and bowels (sites where such effects with subsequent hemorrhages have been observed in neonates), cavitation cannot occur in these organs [[71], [72], [73]]. Although bioeffects have been documented in animal models, this is not the case for humans, especially when an epidemiological approach is used [[71], [72], [73], [74]]. Only non-right handedness is real [75], and even it seems to be more common in male fetuses and to have low statistical significance [74]. It has been suggested, but not proven, that autism has other subtle (as in difficult to diagnose, not as in severity or influence) implications as well [76]. Since the baby is more vulnerable to external insults during organogenesis, which occurs mostly between weeks 10 and 12, of gestation, despite the fact that numerous organs continue to develop later, this is a unique circumstance that arises early in pregnancy [77,78]. This is crucial because endovaginal ultrasonography is increasingly being used in early pregnancy, reproductive endocrinology, and anatomy surveys.

The article "Liability, risks, and recommendations for ultrasound use in the diagnosis of obstetrics diseases" was retracted in 2025. Reasons: unreliable results or conclusions; concerns about the citations.

Doppler ultrasound, especially pulsed (or spectrum), should be used with extreme care. There is a huge disparity between the mean I_SPTAs_ of Bmode (34 mW/cm^2^) and pulsed Doppler (1180 mW/cm^2^). In a previous investigation, on day 19 of a 21-day incubation period, the brains of chicks were subjected *in ovo* to 5 or 10 min of B-mode or to 1, 2, 3, 4, or 5 min of pulsed Doppler ultrasonography, and the results were highly alarming. After hatching, the offspring's cognitive abilities were tested. Memory was unaffected by being exposed to B-mode radiation. However, after 4 and 5 min of exposure to pulsed Doppler, there was a significant impairment of short-, intermediate-, and long-term memory. Furthermore, a second training session did not improve the chicks' performance [79]. This research does raise some worry about possibly subtle impacts of Doppler ultrasonography, however straight extrapolation may not always be true [64,80]. Pulsed Doppler exposure should be minimized in the first trimester [81,82].

### 2.17 Recommendations

The ability to adapt quickly to new developments in medicine, communicate effectively with pregnant women while respecting their autonomy in making decisions, and achieve the highest possible levels of ultrasound performance and detailed reporting of the findings are all crucial to the safety of medical professionals. The person receiving the ultrasound is the one who most cares about maintaining the procedure's safety. It is essential to provide advice supported by solid research, although this might be difficult.

Diagnostic ultrasound should be used sparingly and with minimal exposure only when clinically necessary, according to current guidelines. It is also important to limit how long an object is exposed [83]. Those are the parts that make up the As Low As Reasonably Achievable (ALARA) standard. British Medical Ultrasound Society (BMUS) guidelines are the most stringent available [[84], [85], [86]]. They repeated their 1999 Statement in 2009, which states, “For equipment for which the safety indices are displayed over their full range of values, the TI should always be less than 0.5 and the MI should always be less than 0.3.” [87] A maximum temperature of less than 1 °C and a maximum risk index of less than 0.3 are required when the safety indicators are not shown. Avoiding repeated exposure to the same material is recommended [84,88]. Depending on the TI, they propose a very limited amount of time for exposure [84].

Ultrasound exams provide a small but real danger to the developing embryo and fetus, and should be performed with care in feverish patients. Mechanical phenomena need far less stringent precautions since they are likely to be insignificant when there are no gas nuclei present, as is the situation in a fetus's lungs and intestines (presuming no contrast agents are used, of course). In the early stages of pregnancy, extreme care should be used while using pulsed Doppler [[89], [90], [91]]. While adverse effects have been shown in cell cultures and in experimental animals, people have been using diagnostic ultrasonography for over half a century with no reported negative side effects. Studies in this area would benefit greatly from using a double-blind design, randomly assigning half the population to undergo ultrasound screening and the other half to get no screening at all. This would be very challenging to do in a human population due to the wide variety of prenatal ultrasound referrals that are already made and the high prevalence of diagnostic ultrasound in pregnancy. Given that both TI and MI ignore the passage of time, it is possible that we need new or better indices [92]. While B-mode ultrasound is largely safe when used as medically required, it is still important to exercise care, especially during the first trimester of pregnancy and while using Doppler mode, since there are still some gray areas. If just as much time as is absolutely required to get an accurate picture is spent on the test, M-mode and 3D/4D ultrasonography seem safe (Fig. 1). Keeping ultrasound's good safety record and preventing any negative bioeffects requires diligent end-user education [93].

The article "Liability, risks, and recommendations for ultrasound use in the diagnosis of obstetrics diseases" was retracted in 2025. Reasons: unreliable results or conclusions; concerns about the citations.

**Fig. 1:** Advantages of 4D ultrasound in obstetrics.

Moreover, when conducting an investigation or treatment as part of a research program, or when the treatment or procedure is complex, involves substantial hazards and/or side effects, or may have major implications for the patient's employment, social, or personal life, written consent is required from the patient. If the patient's case records include the pertinent information of the consent conversation, including the patient's particular demands and the nature of the services to which they are agreeing, then oral consent may be accepted. However, regular screening is often administered on an opt-out rather than opt-in basis in hospitals. Since a scan is legally equivalent to a blood test, informed consent is often not recorded. All patients should be offered the option to decline the standard scan without affecting their prenatal treatment, and this should be recorded. Even if a patient's ability to sue a negligent doctor or health care specialist may not be affected by whether or not they gave their informed permission in writing, this document is nevertheless very useful to the defense.

The article "Liability, risks, and recommendations for ultrasound use in the diagnosis of obstetrics diseases" was retracted in 2025. Reasons: unreliable results or conclusions; concerns about the citations.

## 3 Conclusion

Keeping up to date on the latest standards, procedures, and policies is crucial for practitioners conducting and interpreting ultrasound tests, especially in light of the fast developments in ultrasonography expertise and technology. The importance of ultrasonography in contemporary obstetrics and gynecology is that it must be included into routine practice. It might be challenging to determine whether a patient should be sent to a specialist for a more thorough ultrasound assessment. An ultrasound scan may be difficult to interpret, therefore it is important to connect patients to the right specialists. It is crucial to offer and maintain high-quality ultrasound equipment at all diagnostic levels. It is also crucial that employees be certified and that procedures be followed. Periodic retrospective assessments of ultrasound examinations, particularly in situations of misdiagnosis, are recommended as a component of an ongoing quality improvement strategy. Images, video loops, and reports should all be stored safely. Ultrasound testing may be very helpful. Eventually, providers may better manage and educate patients if they are aware of the risks associated with ultrasonography.

## Ethics approval

Not applicable.

## Consent to participate

Not applicable.

## Consent for publication

Not applicable.

## Funding

This study was supported by Xiangshan County Science and technology Project (No. 2022C6013).

## Availability of data and materials

No data was used for the research described in the article.

## CRediT authorship contribution statement

**Haiting Sun:** Conceptualization, Formal analysis, Funding acquisition, Investigation, Resources, Software, Writing – original draft, Writing – review & editing. **An Wu:** Data curation, Formal analysis, Funding acquisition, Investigation, Methodology, Resources, Software, Validation, Visualization, Writing – original draft, Writing – review & editing. **Minli Lu:** Formal analysis, Funding acquisition, Investigation, Methodology, Resources, Software, Validation, Visualization, Writing – original draft, Writing – review & editing. **Shan Cao:** Formal analysis, Funding acquisition, Investigation, Project administration, Software, Supervision, Writing – original draft, Writing – review & editing.

## Declaration of competing interest

The authors declare that they have no known competing financial interests or personal relationships that could have appeared to influence the work reported in this paper.

## List of abbreviations

PUL: Pregnancy of Unknown Location
BMUS: British Medical Ultrasound Society
CPT: Current Procedural Terminology
AIUM: American Institute of Ultrasound in Medicine
ASRM: American Society for Reproductive Medicine
ACOG: American College of Obstetricians and Gynecologists
PACS: picture archiving and communication system
